The article "Determination of Benzalkonium Chloride in a Disinfectant by UV Spectrophotometry and Gas and High-Performance Liquid Chromatography: Validation, Comparison of Characteristics, and Economic Feasibility" was published in 2022. Journal: Int J Anal Chem.

# Determination of Benzalkonium Chloride in a Disinfectant by UV Spectrophotometry and Gas and High-Performance Liquid Chromatography: Validation, Comparison of Characteristics, and Economic Feasibility

**DOI:** 10.1155/2022/2932634

**Published:** 2022-09-19

**Authors:** Mariia Smolinska, Roman Ostapiv, Mariia Yurkevych, Liubov Poliuzhyn, Olha Korobova, Ihor Kotsiumbas, Hryhorii Tesliar

**Affiliations:** State Scientific Research Control Institute of Veterinary Preparations and Fodder Additives, Donetska Str 11, Lviv 79019, Ukraine

## Abstract

Simple, fast, and validated UV-spectrophotometric, HPLC, and GC methods for the analysis of benzalkonium chloride in a disinfectant were developed. UV-spectrophotometric determination was based on measuring the amount of light absorption of aqueous solutions of benzalkonium chloride at 268 nm. HPLC determination was achieved with a 150 mm × 4.6 mm, 5.0 *μ*m C18 column. The mobile phase consisted of a 0.01% water solution of triethylamine (with pH 2.5) and acetonitrile in the ratio of 40 : 60 v/v. The column temperature was kept at 30°C, and the injection volume was 10 *μ*L. The flow rate was 1.0 mL/min, and the diode array detector was set at 215 nm. GC determination was performed using a flame ionization detector on a glass capillary column ZB-WAX plus 30 m × 0.25 mm with an inner coating thickness of 0.25 *μ*m. It creates a gradient increase in the temperature of the furnace to the maximum of 200°C. The temperature of the injector was 250°C, 1 *μ*l was injected, and the separation of the sample was 1 : 100. Helium was used as a carrier gas, and the gas flow rate was constant, equaling 1.6 ml/min. The temperature of the detector was 250°C, and a mixture of hydrogen, helium, and air in a ratio of 30 : 8.5 : 350 was used in the split of the detector. All proposed methods were validated according to ICH guidelines with respect to the accuracy, precision (interday, intraday, and reproducibility), linearity, the limit of detection, the limit of quantitation, and robustness. All three methods were linear (*R*^2^ = 0.997–0.999) over a concentration range of 400–600 *μ*g/ml for UV and 80–120 *μ*g/ml for HPLC and GC, accurate (recovery was 98.4–101.7% for all methods), precise (RSD <2%), and robust. The cost of the analysis of one sample of the disinfectant for the content of benzalkonium chloride by three methods was calculated. The comparison of the obtained results facilitates a more efficient allocation of laboratory resources, depending on the goal.

## 1. Introduction

Benzalkonium chloride (BAC; CAS № 63449-41-2) is a mixture of alkyl dimethyl benzyl ammonium chlorides. They have the common formula [C_6_H_5_CH_2_N(CH_3_)_2_R] Cl, where R is a mixture of alkyls, including all or some of the groups starting with n-С_8_Н_17_, and other higher homologues, such as n-С_12_Н_25_, n-С_14_Н_29_ and n-С_16_Н_33,_ which form the main share (Figure 1) [1]. The average molar mass is 360 g/mol.

The article "Determination of Benzalkonium Chloride in a Disinfectant by UV Spectrophotometry and Gas and High-Performance Liquid Chromatography: Validation, Comparison of Characteristics, and Economic Feasibility" was published in 2022. Journal: Int J Anal Chem.

BAC solutions have antimicrobial activity against a wide range of bacteria, both Gram-positive and Gram-negative, and fungi (being minimally active against bacterial endospores and acid-producing bacteria, relatively inactive—against spores and moldiness, and active against some viruses, including HIV).

ВAС is used in pharmaceuticals as an antimicrobial preservative. It is most widely used in ophthalmic drugs (eye drops and ointments) as well as nasal drops, which are required to produce a rapid bactericidal effect without irritating mucous membranes [2]. It is also known about the use of BAC in drugs for intravaginal use [3–6]. It is used in disinfectants, which have recently proved to be extremely important in the global pandemic for maintaining cleanliness in public places. This is a new challenge for the analysis of control laboratories, as the large number of samples to be analyzed creates additional difficulties. Therefore, a need emerges to use, on the one hand, simple and cheap and, on the other, accurate and correct methods of analysis. Consequently, the aim of our work was to validate and compare the characteristics of three methods—the UV-spectrophotometric (UV) one, the method of high-performance liquid (HPLC), and gas (GC) chromatographies—for their adequate use depending on the object of analysis, laboratory capabilities, and customer needs.

The periodical scientific literature focusing on the determination of BAC offers a spectrophotometric method in its variations—direct [7–9], derivative [10], differential [11, 12] spectrophotometry, and the method of extraction-spectrophotometric determination [13, 14]. The use of the methods of HPLC [15–18], thin-layer [19] and GC [20], chromatography-mass spectrometry [21], capillary electrophoresis [22], and potentiometric titration using ion-selective electrodes for BAC quantitative determination [23] has also been reported. In accordance with the requirements of the European Pharmacopoeia [24] and the British Pharmacopoeia [25], quantification of the basic substance in the BAC substance is performed by two-phase iodometric titration using methylene chloride in EP and chloroform in BP. Following the requirements of the USA Pharmacopoeia [26], quantification is conducted by the HPLC method. There is no article in the State Pharmacopoeia of Ukraine [27] on the BAC substance. Also, none of the pharmacopoeias possess information on the determination of BAC in combined disinfectants.

The article "Determination of Benzalkonium Chloride in a Disinfectant by UV Spectrophotometry and Gas and High-Performance Liquid Chromatography: Validation, Comparison of Characteristics, and Economic Feasibility" was published in 2022. Journal: Int J Anal Chem.

The HPLC and UV are good approaches to detecting aromatic alkylammonium surfactants. GC analysis can be used to determine aromatic surfactants, to which benzalkonium chloride belongs, as evidenced by the work [28]. According to basic research [20, 29], GC-FID is used for the quantitative determination of BAC.

The object of study was the “VIROSAN F” disinfectant—a complex detergent and disinfectant that acts bactericidal. Quantitative determination of BAC in such a disinfectant can be complicated by the influence of glutaral dialdehyde, formaldehyde, and syntanol [30].

Thus, the aim of our work was to develop and validate several methods for determining BAC in the presence of aldehydes (glutaral and formaldehyde) and excipients by the UV method as routine and HPLC or GC as arbitrage to control the quality of generic preparations, since a wide range of methods provides laboratories with more degrees of freedom without reducing their qualification.

## 2. Experiment

### 2.1. Equipments Instrumentation and Software

Laboratory glassware grade A (SIMAX, Czech Republic) and electronic weight AS 220. R2 (“Аxis,” Czech Republic) were used. Bidistilled water was purified by Adrona Crystal EX (Latvia).

A double-beam UV-Visible spectrophotometer (Model UV-2600, Shimadzu, Japan) equipped with wavelength accuracy of +0.5 nm (with automatic wavelength correction) and l cm cuvettes were used. All absorbance measurements were performed at−20°C.

The HPLC analysis was carried out on the “Dionex Ultimate-3000” (Thermo Scientific, USA) equipped with pump LPG-3400SD, autosampler ACC-3000, UV-detector VWD-3100, and LC column Kinetex C18 (150 × 4.6 mm, 5 *μ*m).

The GC analysis was carried out on an HP-6890 Plus gas chromatograph (Hewlett-Packard, USA) equipped with a flame ionization detector and a ZB-WAXplus 30 × 0.25 × 0.25 *μ*m glass capillary column.

The object of analysis was the “VIROSAN F” disinfectant, which contains benzalkonium chloride (50 mg/ml), glutaraldehyde, formaldehyde, syntanol DS-10, and highly purified water. This disinfectant was obtained from a manufacturer [30].

### 2.2. Spectrophotometric Conditions for the Absorption Correction Method

#### 2.2.1. Experimental Condition

The light absorption spectra of the BAC solutions were taken in the range from 220 nm to 300 nm, and the optical density was measured at *λ* = 268 nm in a quartz cuvette with an optical path of 1 cm length using water as a reference solution.

#### 2.2.2. Preparation of Solutions for Spectrophotometric Analysis

A working solution of the standard sample was prepared by dissolving and then diluting 100 mg of BAC (50% solution) in water by 100 times.

The article "Determination of Benzalkonium Chloride in a Disinfectant by UV Spectrophotometry and Gas and High-Performance Liquid Chromatography: Validation, Comparison of Characteristics, and Economic Feasibility" was published in 2022. Journal: Int J Anal Chem.

The model of preparation was produced by mixing the components in a beaker in accordance with the qualitative and quantitative composition as indicated in the manufacturer's documentation. The contents were then quantitatively transferred to a 100 ml volumetric flask, made up to the mark with water, and mixed thoroughly. The working solution was prepared by diluting 1 ml of the model mixture 100 times with water.

The model mixture of placebo was prepared in the same way as the model mixture of the drug, but without adding BAC.

#### 2.2.3. Analysis of Marked Formulation

An aliquot of the preparation containing 100 mg of BAC (2 g of the drug) was dissolved in 30 ml of double-distilled water in a 50 ml volumetric flask, mixed thoroughly, and made up to the mark. 5 ml of this solution were made up to the mark with the same solvent in a volumetric flask with a capacity of 20 ml.

### 2.3. HPLC Studies

#### 2.3.1. Experimental Condition

The mobile phase consisted of the 0.01% water solution of triethylamine (titrated with 1 M NaOH to pH 2.5) and acetonitrile in the ratio of 40 : 60% v/v. A membrane filter of 0.45 *μ*m porosity was used to filter and degas the mobile phase by sonication. Separation was carried out using isocratic elution on LC column Luna C18 (2) 250 × 4.6 with the particles diameter of 5 *μ*m. The flow rate was 1.0 ml/min, and the detector was set at 215 nm. The volume of the sample solution injected was 10 *μ*l. The analysis was conducted at 30°C. As a solvent for the preparation of working solutions, a volumetric mixture of methanol and water in a 1 : 1 ratio was used.

#### 2.3.2. Preparation of Standard Stock and Working Solutions for HPLC Studies

A standard stock solution was prepared by dissolving and then diluting 100 mg of BAC (50% solution) in the 50 ml volumetric flask. A standard working solution was prepared by diluting the standard stock solution by 10 times.

#### 2.3.3. Preparation of Disinfectant Stock and Working Solutions for HPLC Studies

An aliquot of the disinfectant containing 50 mg of BAC (1 g of the disinfectant) was dissolved by a volumetric mixture of methanol and water in a 1 : 1 ratio in the 50 ml volumetric flask (a sample stock solution). A sample working solution was prepared by diluting the sample stock solution 10 times with further filtering through the membrane filter with a 0.45 *μ*m pore diameter.

### 2.4. GC Studies

#### 2.4.1. Experimental Condition

The ZB-WAXplus 30 × 0.25 glass capillary column with an inner coating thickness of 0.25 *μ*m was used for the study. The separation was performed with a gradient of the furnace temperature at 200°C. The injector temperature was 250°C. The injection volume was 1 *μ*l at a flow rate of 1 : 100. Helium was used as a carrier gas. The gas flow rate through the column was 1.6 ml/min, while the detector temperature was 250°C. The mixture of gases used in the detector consisted of hydrogen, helium, and air in the ratio of 30 : 8.5 : 350.

The article "Determination of Benzalkonium Chloride in a Disinfectant by UV Spectrophotometry and Gas and High-Performance Liquid Chromatography: Validation, Comparison of Characteristics, and Economic Feasibility" was published in 2022. Journal: Int J Anal Chem.

#### 2.4.2. Preparation of Standard Stock and Working Solutions for GC Studies

A standard working solution was prepared by dissolving 500 mg of BAC (50% solution) in 50 ml of water in the volumetric flask.

#### 2.4.3. Preparation of Disinfectant Stock and Working Solutions for GC Studies

A sample working solution of the disinfectant containing 50 mg of BAC (1 g of the drug) was dissolved in water in the 50 ml volumetric flask and then filtered through the membrane filter with a 0.45 *μ*m pore diameter.

### 2.5. Validation Methods

The design of experimental method validation was similar to the work of Shah [31]. Method validation for the quantitative determination of BAC was carried out according to ICH Q2R [32], the State Pharmacopoeia of Ukraine 2.0, v. 1 [27], and the European Pharmacopoeia [24] with the following characteristics:

The system suitability (for HPLC and GC) was established to prove that the suitability and reproducibility of the chromatographic system are adequate for performing the analysis. A single set of standard solutions was prepared, as mentioned in the test method, and five replicate injections of the mixed standard preparation were injected and chromatograms were analyzed. The specificity was checked by comparing the absorption spectra of model solutions and solutions of placebos of the selected veterinary drug. The linearity was checked in the range of 80%–120% of the nominal content of BAC in the preparation at 5 points of 80%, 90%, 100%, 110%, and 120% in three parallel determinations. The sensitivity of the analytical method was evaluated by determining the limit of detection (LOD) and limit of quantification (LOQ) using the following equations:

(1) $$\begin{array}{c} LOD=\frac{3,3\cdot \sigma }{S},\\ LOQ=\frac{10\cdot \sigma }{S}, \end{array}$$

where *σ* = standard deviation of the y intercept of the calibration curve (*n* = 6), and *S* = slope of a regression equation.

The robustness was checked by investigating the stability of the working solutions over time. The accuracy and precision were checked by using the data obtained during the study of linearity. The laboratory precision was checked by analyzing the content of BAC in one series of the drug on different days by two analysts.

## 3. Results and Discussion

The method of spectrophotometric determination of BAC is based on the ability of its aqueous solutions to absorb light in the UV region of the spectrum, namely at 257 nm, 262 nm, and 268 nm. As the analytical wavelength, 268 nm was chosen as the closest to the visible region, and the possible effect of the solvent and other components of the drug appeared to be the lowest. Chromatographic studies by HPLC and GC were performed in order to develop an arbitration method for the determination of BAC in this disinfectant and possible analogues. The developed and optimized method was validated for system suitability, specificity, linearity, accuracy, and precision (repeatability and intermediate precision).

The article "Determination of Benzalkonium Chloride in a Disinfectant by UV Spectrophotometry and Gas and High-Performance Liquid Chromatography: Validation, Comparison of Characteristics, and Economic Feasibility" was published in 2022. Journal: Int J Anal Chem.

### 3.1. System Suitability

The standardization for the chromatographic system suitability test was established based on the requirements and FDA recommendations for the liquid chromatography method [27, 33]. System suitability was established to prove that the suitability and reproducibility of the chromatographic system are adequate for performing the analysis. A single set of standard solutions was prepared, as mentioned in the test method, five replicate injections of the mixed standard preparation were injected, and a chromatogram was taken. The results are shown in Table 1.

### 3.2. Specificity

The specificity of the method was determined by comparing the spectra (for UV) and chromatogram (for RP-HPLC and GC-FID) of the standard and sample solutions of BAC. For HPLC, the peak purity index of each compound in the sample solution was found to be nearer to 1. The results obtained under optimized conditions have shown no interference from other common solutions, other active substances (glutaral dialdehyde, formaldehyde), excipients (syntanol), and impurities. The findings demonstrate the specificity of the method (Figure 2).

### 3.3. Solution Stability Study

Solution stability was tested to check whether the BAC was stable in the solvent. The stability test was performed by measuring the absorbance (for UV) and peak area (for HPLC) of the solution at different time intervals. It was observed that BAC was stable in the solution for up to 10 hours at room temperature.

Every three hours, three chromatograms of working solutions were obtained by HPLC and GC, and three spectra were obtained by UV . The results were compared with each other. The solutions were considered stable over time if the value of the found content of BAC did not differ from that for a freshly prepared solution by more than 1.02% (Table 2).

### 3.4. Linearity and Sensitivity

Linearity was investigated within a range of the analytical technique's application. Five solutions were prepared by the dilution of a working solution of the model sample of the drug, with the concentration of BAC ranging from 80% to 120% of its nominal content.

The article "Determination of Benzalkonium Chloride in a Disinfectant by UV Spectrophotometry and Gas and High-Performance Liquid Chromatography: Validation, Comparison of Characteristics, and Economic Feasibility" was published in 2022. Journal: Int J Anal Chem.

Linearity was checked by diluting a standard stock solution at five different concentrations. The linear regression analysis obtained by plotting the absorbance (for UV) and peak area (for HPLC, GC) of analytes vs. concentration has shown correlation coefficients (*R*^*2*^) greater than 0.997. The sensitivity of the analytical method was evaluated by determining LOD and LOQ. The statistical results, such as correlation coefficient, slope, and intercept, are reported in Table 3.

### 3.5. Accuracy

The accuracy of an analytical method is determined by the systemic error involved. Accuracy is the degree of closeness of the test results obtained by this method to the true value. The accuracy of the method was tested at three levels of 80, 100, and 120% of the working concentration of a sample. From the total amount of the compound found, the % recovery rate was calculated. The procedure was repeated three times for each concentration. The % RSD was calculated. The results are shown in Table 4.

### 3.6. Precision

The precision of the method was confirmed by repeatability and intermediate precision. ***Repeatability*** expresses the precision under the same operating conditions over a short interval of time. The repeatability was performed by the analysis of the formulation repeated five times with the same concentration. The amount of each compound present in the formulation was calculated as reported in% RSD. The results for repeatability are shown in Table 5.

The verification of ***intralaboratory precision*** was carried out by a number of analysts who used different dishes and performed 5 parallel measurements for one series of the drug on different days in one laboratory. For all results, a single average value of the content of BAC (m_intra_), relative standard deviation (S_intra_), and relative confidence interval (Δ_intra_) were calculated.

Table 6 shows the results of testing the intralaboratory precision of the method of quantitative determination of BAC in the “VIROSAN F” preparation.

All studies show that the three methods for determining BAC (UV, HPLC, and GC methods) are suitable for controlling the content of this compound in the disinfectant. To effectively allocate the resources of the laboratory, which has facilities to use all three of these methods, we compared the cost (in UAH) of the analysis of one sample of the disinfectant for the content of BAC (HPLC SSCRI laboratory data). The data are provided in Table 7.

These data indicate that it is economically feasible to use the simplest and cheapest method of SF, but only for this specific disinfectant. In other cases, it is likely that other active or auxiliary compounds will affect the analytical signal. It is possible that a change in the components of the disinfectant will change the analytical picture, and in such cases, it will be necessary to use more expensive chromatographic methods.

The article "Determination of Benzalkonium Chloride in a Disinfectant by UV Spectrophotometry and Gas and High-Performance Liquid Chromatography: Validation, Comparison of Characteristics, and Economic Feasibility" was published in 2022. Journal: Int J Anal Chem.

From the point of view of environmental friendliness, the most acceptable is the method of spectrophotometric determination, because its use requires only water —the simplest and most environmentally friendly. The next is the method of gas chromatography, where the solvent is also water. But this method uses a carrier gas mixture of hydrogen, helium, and air, which theoretically can pollute the environment. The most negative impact on the environment may be the method using HPLC method because it is proposed to use a mixture of triethylamine and acetonitrile as a solvent. However, given that the wastewater of analytical laboratories must be purified, any of the proposed methods could be used in industry.

## 4. Conclusion

UV, HPLC, and GC methods were successfully developed and validated for the determination of BAC in the disinfectant. The developed methods were found to be sensitive, accurate, precise, and robust. The results of the assay of the commercial formulation obtained from the UV, HPLC, and GC methods were not significantly different as per the statistical analysis. This implies that the proposed UV, HPLC, and GC methods can be used for quality control analysis of BAC in this disinfectant.

## Figures and Tables

**Figure 1:** Structural formula of BAC (*n* = 8, 10, 12, 14, 16, 18).

**Figure 2:** Electronic absorption spectra and chromatograms of blank (a), standard (b), and sample (c) solutions of the UV (1), HPLC (2), and GC (3) in the determination of BAC.

**Table 1:** System suitability test parameters for BAC by HPLC and GC methods.

Parameters	HPLC				GC			
	Peak 1	Peak 2	Peak 3	Permissible limits	Peak 1	Peak 2	Peak 3	Permissible limits
Retention time, min	4.05	7.69	16.36	—	12.43	13.60	17.28	—
Peak area (% RSD)	0.32	0.40	0.34	≤1.43%	2.44	2.88	2.77	≤1.43%
Tailing factor	1.3	1.4	1.1	0.8 ÷ 1.5	1.06	1.04	1.08	0.8 ÷ 1.5
Theoretical plates	2952	5869	11291	≥2000	3.42 × 10^6^	4.66 × 10^6^	2.23 × 10^6^	≥2000
Resolution factor	10.4	10.4	17.2	≥1.5	8.30	26.10	45.20	≥1.5

**Table 2:** Investigation of the stability of BAC solutions over time.

Parameters	UV	HPLC	GC
	RSD, %		
1 h	0.15	0.30	0.20
2 h	0.29	0.37	0.33
3 h	0.12	0.58	0.47

**Table 3:** Criteria of linearity and sensitivity of BAC determination in the “VIROSAN F”.

Parameters	Value		
	UV	HPLC	GC
*b*	0.001	0.070	5.731
S_*b*_	2.195	0.001	0.245
*a*	−0.029	−0.468	−9.760
S_*a*_	0.011	0.108	24.78
*R * ^*2*^	0.9993	0.9997	0.9973
LOD, (*μ*g·ml^−1^)	29.1	5.1	14.3
LOQ, (*μ*g·ml^−1^)	87.2	15.5	43.2

The article "Determination of Benzalkonium Chloride in a Disinfectant by UV Spectrophotometry and Gas and High-Performance Liquid Chromatography: Validation, Comparison of Characteristics, and Economic Feasibility" was published in 2022. Journal: Int J Anal Chem.

**Table 4:** Criteria of accuracy of BAC determination in the “VIROSAN F”.

Parameters	UV			HPLC			GC		
Level, %	80	100	120	80	100	120	80	100	120
Sample concentration (*μ*g ml^−1^)	400	500	600	80	100	120	80	100	120
Found concentration (*μ*g ml^−1^)	408.6	497.2	602.2	79.2	99.9	122.4	79.4	99.9	121.4
SD	1.43	1.58	1.74	0.06	0.10	0.02	1.70	1.77	1.87
*RSD*, %	0.35	0.32	0.28	0.08	0.10	0.01	0.54	0.42	0.37
Recovery, %	100.7	98.4	99.3	99.0	99.9	102.0	107.2	112.9	111.2

**Table 5:** Test results of the repeatability study of BAC quantitative determination in the “VIROSAN F”.

Parameters	UV	HPLC	GC
M, mg/ml	49.50	48.70	49.07
SD^*∗*^	0.31	0.24	0.98
RSD^*∗*^, %	0.76	0.19	0.28

^*∗*^Mean of 5 determinations.

**Table 6:** Test results of intermediate precision of BAC quantitative determination in the “VIROSAN F”.

Parameters	UV		HPLC		GC	
	1^st^ day	2^nd^ day	1^st^ day	2^nd^ day	1^st^ day	2^nd^ day
Intraday precision						
m_intra_, (mg/ml)	49.70	49.88	48.71	48.30	49.07	48.81
SD_*intra*_^*∗*^	0.16	0.28	0.24	0.82	3.4	1.56
RSD_*intra*_^*∗*^,%	0.75	1.38	0.19	0.22	0.99	0.43

*Interday precision*						
m_inter_, (mg/ml)	49.79		48.51		48.94	
SD_*inter*_^*∗*^	0.22		0.53		2.48	
RSD_*intra*_^*∗*^,%	0.42		0.21		0.71	

^*∗*^Mean of 3 determinations.

**Table 7:** The cost of one analysis of the content of BAC in the “VIROSAN F” disinfectant.

Method	The cost of analysis, UAH
UV	950
HPLC	3500
GC	3200

## Data Availability

The data used to support the findings of this study are available from the corresponding author upon request.
